# Morphometric Approach to Pulp Fibroblast Development in Tooth Germ

**DOI:** 10.1155/2014/836583

**Published:** 2014-06-25

**Authors:** Irina-Draga Căruntu, Sergiu Daniel Săvinescu, Cornelia Amălinei

**Affiliations:** ^1^Department of Morpho-Functional Sciences—Histology, Grigore T. Popa University of Medicine and Pharmacy of Iaşi, 16 University Street, 700115 Iaşi, Romania; ^2^County Service of Forensic Medicine, 1 Vasile Alecsandri Street, 730103 Vaslui, Romania

## Abstract

This paper builds a morphometric framework for the analysis of dental pulp fibroblast evolution during tooth development. We investigated 15 tooth germs (cases) organized, by histological criteria, in three groups corresponding to cap, early bell, and late bell stages, respectively. Each group comprised five cases. The morphometric description used the following parameters: area (*A*), perimeter (*P*)—automatically extracted by a color segmentation technique, and form factor (*FF*)—calculated as 4*πA*/*P* ^2^. The designed framework operated at inter- and intragroup levels. The intergroup analysis quantified the differences between groups, in the sense of a relative distance (RD) adequately defined by mean-value scaling. We showed that the stage of early bell is approximately 5 times closer to late bell than to cap. The quantification procedure required concomitant information about *A*, *P* parameters (as *P versus A* dependences, or *FF* values), whereas the procedure failed for *A* or *P* separately used. The intragroup analysis quantified the similarity of the cases belonging to the same stage. We proved that, unlike the intergroup tests, the individual exploitation of all three descriptors *A*, *P*, and *FF* is effective, yielding highly compatible results. Within any group, most cases presented RDs less than 10% from the group mean value, regardless of the descriptor type.

## 1. Introduction

Dental research papers dealing with the quantitative exploration of the tooth and its specialized supporting tissues are rather scarce, compared with quantitative studies referring to other tissues or organs, in normal and pathological conditions. The papers issued before the late eighties rely on the classical principles of morphometry (i.e., manual identification of the interest regions and grid-based measurements), whereas the more recent works benefit from computer vision facilities in morphometry (i.e., different automation degrees in identification of the interest regions and pixel-level accuracy in measurements). These studies (regardless of the morphometric approach complexity) are almost entirely oriented towards the mature, permanent teeth.

A review of the scientific contributions based on morphometric investigations underlines the main addressed topics. The first papers (using classic morphometric methods) offer data about the differences between deciduous and, respectively, permanent dentition [1], the marginal periodontal tissue [2], and analyze the quantitative changes of the dentin [3–5] and cementum [4], in relationship with the aging process.

Computerized morphometry has rapidly become a valuable tool for the assessment of the tooth and oral tissues. An experimental study [6] quantified the areas of enamel, dentin, and pulp using image analysis morphometry, in parallel with the analysis of the mineralization levels of enamel, dentine, and alveolar bone using quantitative microradiography and a microphotometric-microdensitometric technique. Other studies dedicated to the evaluation of dentin sizes, according to biological age, are realized [7].

The human dental pulp is a central subject, in terms of the quantitative information related to the odontoblasts [8, 9], to the immune cells present in deciduous and permanent tooth, in normal status and disease [9–11], and to the nervous elements [12]. Another interesting idea is represented by the quantitative analysis on the influence of over retention on the oral and pulp tissues of human primary teeth. In the pathology field, there are some results on the quantitative morphological changes in periapical lesions [13, 14], the histopathological and immunofluorescence exams being correlated with the radiological aspects [15], as well as on the collagen dynamic in dentin carious lesions [16].

The aim of our work is to study the quantitative features of fibroblasts, during tooth development. In accordance with the literature overview briefly presented above, investigations on this topic are completely absent, a fact which motivates our research and concomitantly ensures the novelty of the results. A key issue addressed here is the role of morphometry in detecting the differences between the development stages,* strictly referring* to dental papilla or pulp, respectively, which is a rather difficult task for the visual capacity of human observers. Thus, our study provides a morphometric profile for the evolving fibroblasts, in order to complement the classic qualitative knowledge about the development stages, by quantitative information that is able to refine the characterization of the dental papilla and dental pulp.

## 2. Material and Methods

### 2.1. Tissue Procurement and Processing

The study material included human tissues corresponding to 20 cases, represented by embryos and fetuses with a gestational age of minimum 2 months, collected from medical or spontaneous abortions, and newborns deceased at birth, investigated in the County Service of Forensic Medicine Vaslui and in the Pathology Laboratory of the Municipal Hospital Barlad. Gestational age of each embryo and fetus was established in accordance with maternal records (2 cases—8 weeks, 3 cases—10 weeks, 3 cases—14 weeks, 1 case—16 weeks, 2 cases—18 weeks, 3 cases—22 weeks, 4 cases—24 weeks, and 2 cases—40 weeks). Legal harvesting, manipulation, and conservation conditions were respected, with the collecting of the specimens being performed only with the written consent of the family and certified by an informed consent protocol. The study was approved by the Ethical Committee of the “Grigore T. Popa” University of Medicine and Pharmacy, in accordance with the Helsinki Declaration.

The embryos were fixed in 10% neutral buffered formalin and fully embedded in paraffin, and 4 *μ*m thick serial sections were cut. The cephalic extremities (fetuses aged from 10 to 16 weeks) and the maxillas and mandibles (fetuses aged from 18 to 40 weeks) were carefully removed and, respectively, dissected, fixed in 10% neutral buffered formalin and decalcified in 5% formic acid and 5 g sodium citrate. The decalcification time was variable (minimum 3 days, maximum 3 weeks), depending on the gestational age and, implicitly, on the mineralization degree. After demineralization, the fragments were routinely processed before embedding in paraffin. Finally, serial cross sections were made in 4 *μ*m thickness. All sections were stained with haematoxylin and eosin (HE) staining and analysed by standard histological examination.

Our study focused on the evaluation of the fibroblastic cell population present in mandibular central incisors. From the total number of 29 tooth germs (6 in cap stage, 6 in early bell stage, and 14 in late bell stage) identified as mandibular central incisors through microscopical examination, we have selected 15 (5 cases in each stage) which were used for the development of our research. The selection relied on the quality of the histological images, so as to ensure the relevance of both biomedical information (necessary for the qualitative analysis, also including stage assessment) and numerical information (necessary for the quantitative analysis).

Consequently, the material was organized in 3 groups of study as follows: group I included 5 tooth germs in cap stage (gestational age 10th week i.u.), group II included 5 tooth germs in early bell stage (gestational age 14th–18th week i.u.), and group III included 5 tooth germs in late bell stage (gestational age 22nd–24th week i.u.). Each tooth germ defined a case of our study; the germs (equivalently cases) belonging to a group were labeled from 1 to 5.

### 2.2. Computer-Assisted Procedures

The computerized quantitative analysis was performed in the Zeiss KS400 software [17].

The material for the computerized quantitative analysis comprised digital images of the most meaningful zones of dental papilla/dental pulp, captured with the video camera of a Zeiss microscope. For each case belonging to a given group, 5 images (at ×200 magnification) were acquired in the RGB format, from the serial sections. In the remainder of our paper, these images are referred to as “original images.” By using the automated image-processing techniques (detailed below), all pulp fibroblasts were identified on each image, and the following morphometric features/parameters were measured: area (*A*), perimeter (*P*) and form factor (*FF* = 4*πA*/*P* ^2^) [17]. The results of the measurements were separately stored for each case, meaning about 500–700 records per case. Next, for each case exactly 100 records were randomly selected in order to define the sample vectors for *A*, *P*, and *FF* (each of size 100).

We have designed and implemented three KS400 macros (IMAGMEAS—image measurement, CASESTAT—case statistics, and GROUSTAT—group statistics) that allow the automation of cell measurements, as well as the computation and graphical plotting of the statistical information derived from the measurement results.

The IMAGMEAS macro operates at the level of a single image; it identifies all the cells in the image and extracts and memorizes their numerical features (*A*, *P*, and *FF*).

Any original image (e.g., Figure 1) is preprocessed for increasing the contrast of pulp fibroblasts relative to the extracellular matrix. Then a threshold segmentation technique is applied with appropriate values for the three channels RGB, which yields the separation of regions occupied by the fibroblasts. The result is a binary image from which the regions with very small areas are removed (as being considered scrap), such that the remaining white zones correspond to the fibroblastic cells in the original image (e.g., compare Figures 1 and 2).

The measurements of *A* and *P* are performed for each white region of the binary image by using the KS400 field-feature routines FLDAREA and FLDPERIM, respectively [17]. For each white region the descriptor *FF* is computed; it has a subunitary value that expresses a deformation degree from the ideal case (*FF* = 1) of a geometric form with the smallest perimeter corresponding to a given area (i.e., the lower *FF*, the longer perimeter for the same area).

All values *A*, *P*, and *FF* obtained from an image are written in a database associated with the tooth germ (case) which the image belongs to. The database of a case is completely loaded after the iterative call of IMAGMEAS for the 5 images previously acquired for that case.

The CASESTAT macro operates at the level of a case and provides a characterization of the case in statistical terms. It randomly reads 100 records from the data base loaded by the iterative call of IMAGMEAS, which is equivalent to the random selection of 100 fibroblast cells from the 5 original images available for the case. Thus, the vector samples of *A*, *P*, and *FF* are constructed with the same size (100) for all the 15 cases under study.

For any case, CASESTAT computes mean value and standard deviation and extreme values (min, max) for *A*, *P*, and *FF*.

The GROUSTAT macro operates at the level of a group, returning statistical information and graphic plots that portray the analyzed group. It processes the numerical information available for the five cases belonging to a group, the size of the *A*, *P*, and *FF* vectors being 500. GROUSTAT computes for a group the same parameter as CASESTAT calculates for a case. It also plots the histograms of *A*, *P*, and *FF* organized in 20 classes, each class corresponding to 3.5 *μ*m^2^ on the *A* histogram (Figures 3(a), 3(b), and 3(c)), 7 *μ*m on the *P* histogram (Figures 4(a), 4(b), and 4(c)) and 0.05 on the *FF* histogram (Figures 5(a), 5(b), and 5(c)). The linear regression *P versus A* is studied, accompanied by the visual support of the group scattergram that includes the regression line (Figures 6(a), 6(b), and 6(c)).

### 2.3. Data Analysis

*(a) Statistical Tests.* For the intergroup statistical analysis of the morphometric features (i.e., analysis between the three groups), the ANOVA one-way test was applied by the help of the MATLAB function* anova1 *[18]. A supplementary confirmation was proposed for these tests because, rigorously speaking, the ANOVA assumption on equal variance is slightly violated. For this purpose, we have used the MATLAB function* ttest2* [18], which performs the Student's *t*-test under the assumption of equal or unequal population variances. The *p* value was considered significant for *p* ≤ 0.05, highly significant for *p* ≤ 0.01, and very highly significant for *p* ≤ 0.001. The statistical analysis was also applied for intragroup investigations (i.e., between the cases belonging to the same group), but the intergroup and intragroup objectives were different (as commented in the Discussion section).

*(b) Mean-Value-Scaled Relative Distances (Abbreviated as RDs)*. The characterization of cases and, respectively, groups by the morphometric parameter mean values allows the quantification of the* similarity of the cases within a group* and, respectively, of the* differences between the three groups within the study*. Two quantification procedures can be defined by relying on a single mathematical support that is explained below.

Let *E* = {*e*_1_,…, *e*_*n*_} be a set of *n* elements and denote by *M*(*E*) their mean value; that is, *M*(*E*) = (*e*_1_ + ⋯+*e*_*n*_)/*n*. Introduce the transformation ${\overset{-}{e}}_{i}=(e_{i}-M(E))/M(E)=\left(e_{i}/M(E)\right)-1$, *i* = 1,…, *n*, and define the functions as follows:

- $\text{R}{\text{D}}_{E}(e_{i})=|{\overset{-}{e}}_{i}|=\left|e_{i}-M(E)\right|/M(E)$, which is called the relative distance between *e*_*i*_ ∈ *E* and *M*(*E*),
- $\text{RD}(e_{i},e_{j})=|{\overset{-}{e}}_{i}-{\overset{-}{e}}_{j}|=\left|e_{i}-e_{j}\right|/M(E)$, which is called the relative distance between *e*_*i*_, *e*_*j*_ ∈ *E*.

In these forms, the numerator |*e*_*i*_ − *M*(*E*)| or |*e*_*i*_ − *e*_*j*_| preserves the information about the distances between the initial values. At the same time, the denominator *M*(*E*) means a scaling operation that ensures the independence with respect to the concrete range of the initial values *e*_*i*_, *i* = 1,…, *n*.

In our research we used the function RD_*E*_(*e*_*i*_) for the intragroup analysis and the function RD(*e*_*i*_, *e*_*j*_) for the intergroup analysis.

The function RD_*E*_(*e*_*i*_) measures/expresses the proximity of any element of the set *E* to *M*(*E*). Reasonably small values for all RD_*E*_(*e*_*i*_), *e*_*i*_ ∈ *E*, *i* = 1,…, *n*, reflect a similarity between all the elements composing the set *E*.

The function RD(*e*_*i*_, *e*_*j*_) measures/expresses the proximity of any two elements of the set *E*. Let *e*_*i*_, *e*_*j*_, *e*_*k*_ ∈ *E* be three arbitrary elements of *E*. If RD(*e*_*i*_, *e*_*j*_) is much larger than RD(*e*_*j*_, *e*_*k*_), we conclude that *e*_*j*_ is much closer to *e*_*k*_ than to *e*_*i*_; if RD(*e*_*i*_, *e*_*j*_) and RD(*e*_*j*_, *e*_*k*_) are rather equal, we conclude that *e*_*j*_ is as close to *e*_*k*_ than to *e*_*i*_.

At the* intragroup* level, a set of type *E* was defined for each group (I, II, and III) and for each morphometric parameter (*A*, *P*, or *FF*). Such a set comprises five elements corresponding to the mean values of the five cases belonging to the considered group (and corresponding to the parameters *A*, *P*, or *FF*). Thus, we can calculate the relative distances:

- for intragroup I analysis, RD_g  I_*A*_(*e*_*i*_), RD_g  I_*P*_(*e*_*i*_), RD_g  I_*FF*_(*e*_*i*_), *i* = 1,…, 5 cases in group I;
- for intragroup II analysis, RD_g  II_*A*_(*e*_*i*_), RD_g  II_*P*_(*e*_*i*_), RD_g  II_*FF*_(*e*_*i*_), *i* = 1,…, 5 cases in group II;
- for intragroup III analysis, RD_gIII_*A*_(*e*_*i*_), RD_g  III_*P*_(*e*_*i*_), RD_g  III_*FF*_(*e*_*i*_), *i* = 1,…, 5 cases in group III.

In the* intergroup* analysis, a set of type *E* was defined for each morphometric parameter (*A*, *P*, or *FF*) and comprises three elements corresponding to the mean values of the three groups investigated in our study. Thus, we can calculate the relative distances:

- between groups I and II, RD_*A*_(gI, gII), RD_*P*_(gI, gII), RD_*FF*_(gI, gII);
- between groups II and III, RD_*A*_(gII, gIII), RD_*P*_(gII, gIII), RD_*FF*_(gII, gIII).

## 3. Results

The morphometric profiles of the cases belonging to groups I, II and III are summarized in Tables 1, 2, and 3, respectively. All these tables have the same organization, namely, (i) three similar column blocks are used for the three morphometric parameters *A*, *P* and, *FF*; (ii) the first five entries correspond to the five component cases; (iii) each case entry allocates two rows (the first row displays statistical information and the second one provides the relative distance from the group mean value expressed as a percentage); (iv) the last entry contains a single row that displays statistical information referring to the whole group.

### 3.1. Statistical Tests

*Between any two groups*, the statistical differences were very highly significant (*p* < 0.001), for *A*, *P* and, *FF* vectors.

At the* intragroup level,* the statistical analysis revealed significant differences (*p* < 0.05), for some pairs of cases as follows: group I (*A* vectors, 1*vs*2, 1*vs*3, 2*vs*4, 2*vs*5, 3*vs*4, 3*vs*5; *P* vectors, 1*vs*2, 2*vs*4; *FF* vectors, 1*vs*4, 2*vs*4, 3*vs*4); group II (*FF* vectors, 1*vs*4, 4*vs*5, 2*vs*5, 3*vs*5); and group III (*A* vectors, 2*vs*4, 3*vs*4, 3*vs*5; *FF* vectors, 2*vs*3, 2*vs*5). The abbreviation* vs* is used for* versus*.

### 3.2. Mean-Value-Scaled Relative Distances

The RDs of any case from the mean value of the group which the case belongs to were provided by Tables 1, 2, and 3 (as explained above, in the presentation of those tables).

The RDs between the groups were calculated for each descriptor *A*, *P*, *FF*, by using the information in the last entry of Tables 1–3 (i.e., the mean values of the groups I, II, and III) and yielded the following results: expressed as percentages from the global mean of each descriptor:

- RD_*A*_(gI, gII) = 29.45%, RD_*A*_(gII, gIII) = 30.12%, from the *A* global mean (25.24 *μ*m^2^);
- RD_*P*_(gI, gII) = 43.97%, RD_*P*_(gII, gIII) = 30.71%, from the *P* global mean (49.59 *μ*m);
- RD_*FF*_(gI, gII) = 88.29%, RD_*FF*_ (gII, gIII) = 16.57%, from the *FF* global mean (0.176).

### 3.3. Regression Analysis

For each group we analyzed the linear regression *P versus A* and we obtained the regression equations and the correlation factors reproduced below:

- group I: *P* = 1.4263 *A* + 4.6868; *A*-*P* correlation factor = 0.9023;
- group II: *P* = 1.6758 *A* + 9.5794; *A*-*P* correlation factor = 0.9104;
- group III: *P* = 1.7626 *A* + 9.2303; *A*-*P* correlation factor = 0.8825.

### 3.4. Graphical Plots

The construction of *A* histograms (Figures 3(a), 3(b), and 3(c)), *P* histograms (Figures 4(a), 4(b), and 4(c)), and *FF* histograms (Figures 5(a), 5(b), and 5(c)) allowed a facile analysis of the differences between the fibroblastic populations in the three groups. Each histogram was complemented by a graphical plot of the Gaussian distribution with the same mean value and standard deviation of the empirical variable.

The scattergrams *P versus A* corresponding to groups I, II, and III were plotted in Figures 6(a), 6(b), and 6(c). We considered the same ranges for the scattergram axes in order to simplify the visual interpretation of the similarities and differences between the populations of the three groups from the point of view of the cell dimensions. Figures 6(a), 6(b), and 6(c) also depict the regression lines corresponding to the three equations given above. For a complete understanding of the differences between the regression equations associated with the three groups, Figure 7 presents a comparative plot of the three regression lines.

## 4. Discussion

### 4.1. Noticeable Trends in Fibroblast Research: Scarce Morphometric Support

The pulp fibroblasts represent a class of fibroblast population characterized by a high degree of heterogeneity. Their functional potential is extremely large, from the inductive role in tooth development to the repair function typical to mature teeth. In the successive stages of tooth development, the young fibroblasts organized as dental papilla and, later on, as dental pulp contribute to the differentiation of oral epithelium and induce the formation and evolution of the enamel organ. These processes are possible through a cascade of molecular mechanisms, generically named epithelio-mesenchymal interactions [19, 20]. For the mature tooth, the fibroblast involvement in the pulp and dentin repair is a fact unanimously accepted [21–25]. Numerous studies* in vivo* and mainly* in vitro* have proved the effect of several growth factors on the multiplication of dental pulp fibroblasts [26–29], an action that can be continued, if necessary, by their transformation into odontoblasts [30, 31].

An overview of the literature revealed the absence of studies on the quantitative features of fibroblasts* during the tooth development*. The morphometric approach of the fibroblastic population is limited to two studies that refer to the repair function of dental pulp [32, 33], the former was performed on human material, whereas the latter on animals. Both studies analyzed the mature dental pulp, and the purpose was to assess the changes of the cellular density (odontoblasts, subodontoblasts, and fibroblasts) of the pulp total area and of the width of dentin, in correlation with the biological age. The results show that the patient aging implies the increase of dentinal thickness and the decrease of the density of odontoblasts, subodontoblasts, and pulp fibroblasts, both in the crown and root regions. These changes are asymmetrical and more prominent at the root level than in the crown. The two papers indicate that the decrease in pulp cell density may reduce the pulp repair activity, although the increase in dentinal thickness may aid in the pulp protection.

### 4.2. Progress in Fibroblast Research via Morphometry

The investigation of fibroblasts during the tooth development is the key element that ensures the individuality of our work within the context of dental morphometry researches reported in the literature.

Our investigation is founded on a quantitative point of view carefully built from relevant measurement results, which permits a deeper understanding of the fibroblast evolution in connection with tooth development stages. In other words, our mathematical-type findings (i.e., statistical characterizations of the *A*, *P*, *FF* features for the three groups, corresponding to the cap, early bell, and late bell stage, resp.) offer new and irrefutable support for an approach complementary to the traditional analysis based on the qualitative observations of cell transformation (i.e., size and shape modifications).

Thus, the results presented by the previous section yield the following remarks, structured on intergroup and intragroup levels.

#### 4.2.1. Key Points in Intergroup Analysis

(i) The very highly significant differences between the *A* vectors (resp., *P* vectors) of any two groups are in full accordance with the class organization (cap, early bell, and late bell stages) used in the tooth development. Actually, the literature does not discuss the statistical aspects of the morphometric features in fibroblast evolution relative to this class organization. It is important to notice that the* statistical difference* (exclusively referring to the morphometric features of the fibroblasts) between the groups is in full accordance with the* histological difference* (referring to the tooth germs, as complete entities) between those groups. This accordance is explained by the inherent involvement of the morphometric features in the growing process. For such processes, the separation in several groups from histological criteria would be questionable in the absence of statistically significant differences for some morphometric features.

(ii) If the histograms of the *A* vectors (resp., *P* vectors) in Figures 3(a), 3(b), and 3(c) (resp., Figures 4(a), 4(b), and 4(c)) are sequentially analyzed, from group I to group III, then we can say that the numerical interval (mean − standard deviation, mean + standard deviation) for the *A* feature (resp., *P* feature) “moves” from left to right. For a concrete discussion, we also use the values in the last rows of Tables 1–3 and we find the following: (i) for the *A* feature, [10.4, 25.05] *μ*m^2^ (group I) → [14.8, 35.5] (group II) → [21.6, 43.9] (group III) and (ii) for the *P* feature, [18.3, 41.5] *μ*m (group I) → [32.7, 70.8] (group II)→ [44.8, 89.2] (group III).

For each group, the *A* histogram (resp., *P* histogram) shows that the above *A* interval (resp., *P* interval) includes about 350 cases (i.e., approximately 70% from the population, which is rather close to the percentage guaranteed by the ideal Gaussian distribution for the same type of intervals).

The preponderant location of the *A* and *P* features within the aforementioned intervals is also reflected by the scattergrams in Figures 6(a), 6(b), and 6(c), where the *A* intervals move left to right, and the *P* intervals move bottom-up (when comparing the three groups, from I to III). Thus, we got a nice confirmation, exclusively relying on morphometric arguments, for the fibroblast growing process (from the cap to the early bell and, respectively, late bell stage), which is thoroughly described in tooth histology but without numerical information.

(iii) Besides the dimension features (*A* and *P*), the *FF* feature is also involved in the analysis of the fibroblast evolution. Tables 1–3 show that the mean value of *FF* decreases from 0.28 (group I) to 0.13 (group II) and to 0.10 (group III). These values quantify important changes for the cell shapes in the sense that the ratio (perimeter/area-unit) increases from group I to group III. As an example, if we consider three cells with the same area belonging to groups I, II and III, respectively, then the cell in group I has the smallest perimeter, the cell in group III has the greatest perimeter, and the perimeter of the cell in group II has an intermediate value. This increase of the perimeters (while areas are preserved) may be explained by elongation typical to the fibroblast evolution towards fibrocyte. Subsequently, the *FF* values determined for the three groups can be regarded as measures of the modifications in the cell shape, from star-like (in cap stage) to almost fusiform (in late bell stage). It is worth noting the refined action of *FF* as a shape-change measure which is able to reveal that the modifications from group I to II (0.28 to 0.13 mean values) are more significant than the modifications from group II to III (0.13 to 0.10 mean values). The mean values give a significant, but punctual description of the discussed modifications between groups. A global picture is offered by the three histograms in Figure 5, where the plots Figures 5(b) and 5(c) have similar silhouettes, while plot Figure 5(a) differs drastically. This remark has a solid motivation in descriptive tooth biology, in the sense that cap and bell are stages completely separated (involving major differences), whereas early and late bells are phases of the same stage (involving smaller differences).

(iv) Another morphometric proof that the early bell stage is much closer to the late bell stage than to the cap stage results from the comparison of the values calculated for RDs between the groups, with respect to *FF* (16.57% between groups II and III unlike 88.29% between groups I and II). Note that the ratio of the two RDs is 0.8829/0.1657 = 5.3283. At the same time, the RDs with respect to *A* (30.12% between groups II and III and 29.45% between groups I and II) or *P* (30.71% between groups II and III and 43.97% between groups I and II) are unable to give such information. The mathematical merit of these relative distances consists in the robustness with respect to the concrete size of the examined fibroblasts (due to the *M*(*E*) scaling used in the definition of the RD(*e*_*i*_, *e*_*j*_) function; see “Material and Method” section). In other words, for experiments on new groups we expect intergroup relative distances with values similar to this study, regardless of the inherent biological variation of the dimensions (possibly reflected by significantly different mean values for *A*, *P*, and *FF*).

(v) The above paragraph shows that the separate use of information on *A* or *P* cannot quantify the intergroup differences, whereas the *FF* information can do this. Since the definition of *FF* parameter combines the two parameters *A*, *P*, we are motivated to investigate the capabilities of *P versus A* dependences. We use the regression equations and the graphical plot in Figure 7 presented in the “Results” section. It is obvious that the regression line of group II is much closer to the regression line of group III than to the regression line of group I. In numerical terms, if we select the value *A* = 30 *μ*m^2^ (around which there exist many measured values within each of the three groups), then the *P* values on the three regression lines are *P*_I_ = 47.4758 *μ*m, *P*_II_ = 59.8534 *μ*m, and *P*_III_ = 62.1083 *μ*m, respectively. The distance between *P*_I_ and *P*_II_ is 5.4892 times greater than the distance between *P*_II_ and *P*_III_. Notice the good concordance between the values 5.4892 and 5.3283, the ratio between the relative distances with respect to *FF* calculated in the previous paragraph.

#### 4.2.2. Key Points in Intragroup Analysis

(i) The existence of the statistical differences between some cases within the same group seems surprising, if the understanding of the case similarity is confined to the similarity of the morphometric parameters. As a matter of fact, this is a severe limitation because in a normal perspective the biological variety is assumed to exhibit morphometrical differences (even if the group is defined in rather strict histological terms). In principle, the fundamental reason for the association of several cases within a group is the histological profile of cells and structures, which does not necessarily involve the same numerical ranges for all classes with respect to the morphometric features. Therefore, we consider that the use of statistical tests at the intragroup level is not relevant. Our research had a precise motivation for using these tests in order to prove that human-coordinated selection of cases belonging to a group may ignore such differences (if any).

On the other hand, the instrument of relative distance proposed in our work is able to explain why the differences discussed above may be ignored. Thus, the variations of the case mean values around the group mean values (in the sense of RDs) can be globally described as follows, by using a realistic threshold of 10%:

 (a) group I
  1. *A* parameter: three cases below 10%; maximum 17.47% for case 2;
  2. *P* parameter: all cases below 10%; maximum 7.56% for case 2;
  3. *FF* parameter: four cases below 10%; maximum 13.29% for case 4;
 (b) group II
  1. *A* parameter: all cases below 10%; maximum 3.87% for case 2;
  2. *P* parameter: all cases below 10%; maximum 3.74% for case 1;
  3. *FF* parameter: three cases below 10%; maximum 10.44% for case 4;
 (c) group III
  1. *A* parameter: all cases below 10%; maximum 6.12% for case 3;
  2. *P* parameter: all cases below 10%; maximum 4.42% for case 3;
  3. *FF* parameter: all cases below 10%; maximum 9.06% for case 4.

It is obvious that, for each group and for each morphometric parameter, most of the cases present variations less than 10% with respect to the group mean value. We have chosen the threshold of 10% since it represents a reasonable limit for the human capacity of accepting intragroup similarities.

(ii) The scattergrams *P versus A* in Figures 6(a), 6(b), and 6(c) also include the regression lines corresponding to the linear equations given in the “Results” section (and already used in the previous subsection). At first glance, a quasilinear dependence between *P* and *A* is disputable, because *P* and *A* have different variations with respect to a variable expressing length. (For instance, if we consider six squares with edges 1, 2, 3, 4, 5, 6, then the variation of *P* means 4, 8, 12, 16, 20, 24, whereas the variation of *A* means 1, 4, 9, 16, 25, 36. In the considered situation, it is obvious that the dependence of the *P* sequence on the *A* sequence is far from linearity.) A deeper insight into the geometry of the fibroblasts belonging to a group reveals that a quasilinear dependence between the *P* vector and the *A* vector is natural. Generally speaking, cells with different sizes do not have the same shape, a fact already commented in connection with the *FF* feature for different groups. As a rule of thumb, we may say that the larger A, the smaller *FF*, meaning that for increasing *A*, the values of *P* ($P=\sqrt{4\pi A/FF}$) are increasing quasilinearly.

### 4.3. Brief Comments on the Morphometric Tools

The approach proposed in this work for the analysis of evolving fibroblasts is founded on our experience in computerized morphometry [34, 35]. The technique used [35] has been considerably improved in order to process large sets of digital images in relatively short time intervals. The segmentation strategy [35] was replaced by a fully automated procedure, based on color segmentation, which is able to operate successfully on all considered specimens, once their staining differs within reasonable limits, predefined in RGB terms. Thus, during several work sessions, we could extract the morphometric features for more than 8,000 cells (from which 1,500 cells were randomly selected for the development of the study).

The principles we relied on in the design and implementation of our morphometric tools can be transferred* mutatis mutandis *to investigations focusing on other types of cells or structures belonging to the tooth, provided that the staining allows a robust identification based on colour properties. It is worth also mentioning that the Zeiss KS400 technology is not compulsory; we preferred it because of our extensive experience with the system, but other software environments can be equally exploited for such applications.

All the above remarks show that our morphometric construction can serve as a basic and flexible guide for researchers interested in addressing morphometry problems in the complex domain of oral biology.

### 4.4. Final Remarks

The initiation and development of this research were motivated by our conviction that a morphometric study of fibroblast during tooth growth might complement the classical, mainly descriptive approach by providing valuable numerical information. To cover the complexity of the proposed study, the morphometric analysis was separately designed for intergroup and intragroup levels. Our key objective was to provide meaningful quantitative criteria for testing the differences between the evolutive stages (intergroup analysis) and the similarities of the cases belonging to the same stage (intragroup analysis).

The effectiveness of the intergroup analysis was ensured through the combined (concomitant) use of the geometric features area (*A*) and perimeter (*P*). The basic idea consisted in the characterization of each stage (group) by its (*P*, *A*) pairs, which defines the *P versus A* dependence of that stage, and, respectively, the set of form factor (*FF*) values corresponding to that stage. The *P versus A* dependences were exploited via the regression lines that encapsulate the fundamental information but are much simpler to handle than the original dependences. The *FF* value sets were exploited via the mean-value-scaled relative distances. Thus, we devised two procedures that quantify the proximity between the three evolutive stages. The procedure based on the regression lines (resp., on the relative distances with respect to *FF*) showed that early bell is 5.48 (resp., 5.32) times closer to late bell than to cap. In parallel, we also proved that the procedure based on the relative distances applied with respect to either *A* or *P* descriptor fails in the interstage quantitative discrimination.

The intragroup analysis also exploited the instrument of relative distances but in the sense of similarity evaluation through the variations of the case mean values around the group mean value. Tests were performed with respect to all three parameters *A*, *P*, *FF*, and for a criterion of 10% variation; the great majority of the tests passed. It is worth noting that the threshold of 10% appearing in our criterion tries to simulate the human frontier between the acceptance and rejection of region similarities, based on comparisons of areas, perimeters, and contour types.

The following facts deserve supplementary comments as relevant issues in our morphometric construction. The *FF* descriptor is able to quantify shape changes and therefore relative distances with respect to this descriptor are reliable tools for testing both intergroup differences and intragroup similarities. Therefore, for the sake of uniformity, one could limit the complete investigation (intra- and intergroup) to the exploitation of *FF* information. Although possible, such a limitation is not recommended because the existence of several procedures for the same criterion (referring either to differences or to similarities) increases the robustness of the tests.

## Figures and Tables

**Figure 1:** Dental pulp fibroblasts: sample from the set of color images acquired for this work.

**Figure 2:** Identification of fibroblast regions: result of color segmentation technique applied to sample image in Figure 1.

**Figure 3:** Histograms of *A* (area) variable for the three groups: (a) group I, (b) group II, and (c) group III.

**Figure 4:** Histograms of *P* (perimeter) variable for the three groups: (a) group I, (b) group II, and (c) group III.

**Figure 5:** Histograms of *FF* (form factor) variable for the three groups: (a) group I, (b) group II, and (c) group III.

**Figure 6:** Scattergrams *P* (perimeter)* versus A* (area) and the corresponding regression lines for the three groups: (a) group I, (b) group II, and (c) group III.

**Figure 7:** Comparative plot of the three corresponding regression lines to group I (dashed), group II (solid), and group III (dashdot).

**Table 1:** Morphometric characterization of group I.

Case	Area *A* (*μ*m^2^)			Perimeter *P* (*μ*m)			Form factor *FF*		
	Mean ± SD RD_gI_*A*_ (%)	Min	Max	(Mean ± SD) RD_gI_*P*_ (%)	Min	Max	(Mean ± SD) RD_gI_*FF*_ (%)	Min	Max
1	18.755 ± 7.549 5.7%	7.129	35.550	31.582 ± 11.844 5.3%	13.264	59.180	0.272 ± 0.114 5.9%	0.099	0.592
2	14.635 ± 5.903 17%	5.078	30.698	27.712 ± 10.178 7.5%	10.568	63.837	0.271 ± 0.111 6.4%	0.090	0.742
3	16.356 ± 7.202 7.7%	5.317	35.065	29.281 ± 11.222 2.3%	11.802	59.420	0.273 ± 0.113 5.7%	0.109	0.606
4	20.335 ± 7.730 14%	8.556	43.034	31.170 ± 13.122 3.9%	11.082	73.705	0.328 ± 0.161 13%	0.089	0.891
5	18.558 ± 6.855 4.8%	7.530	37.958	30.154 ± 11.168 0.5%	11.887	65.114	0.303 ± 0.137 4.8%	0.082	0.769
Group I	17.733 ± 7.328	5.078	43.034	29.980 ± 11.585	10.568	73.705	0.289 ± 0.130	0.082	0.891

**Table 2:** Morphometric characterization of group II.

Case	Area *A* (*μ*m^2^)			Perimeter *P* (*μ*m)			Form factor *FF*		
	Mean ± SD RD_gII_*A*_ (%)	Min	Max	(Mean ± SD) RD_gII_*P*_ (%)	Min	Max	(Mean ± SD) RD_gII_*FF*_ (%)	Min	Max
1	26.058 ± 10.620 3.4%	8.861	52.743	51.903 ± 20.556 0.2%	20.347	117.308	0.143 ± 0.064 6.8%	0.032	0.371
2	24.212 ± 10.647 3.8%	7.351	50.952	51.065 ± 18.990 1.4%	20.127	98.376	0.129 ± 0.049 3.2%	0.047	0.285
3	25.629 ± 10.629 1.7%	9.159	54.173	52.892 ± 19.011 2.1%	19.448	99.785	0.129 ± 0.053 3.5%	0.052	0.351
4	24.499 ± 10.562 2.7%	7.746	53.395	53.228 ± 19.847 2.7%	22.611	106.470	0.120 ± 0.042 10.4%	0.053	0.219
5	25.538 ± 9.320 1.3%	9.027	58.368	49.854 ± 16.851 3.7%	18.370	97.057	0.147 ± 0.063 10.2%	0.054	0.344
Group II	25.187 ± 10.351	7.351	58.368	51.788 ± 19.055	18.370	117.308	0.134 ± 0.056	0.032	0.371

**Table 3:** Morphometric characterization of group III.

Case	Area *A* (*μ*m^2^)			Perimeter *P* (*μ*m)			Form factor *FF*		
	Mean ± SD RD_gIII_*A*_ (%)	Min	Max	(Mean ± SD) RD_gIII_*P*_ (%)	Min	Max	(Mean ± SD) RD_gIII_*FF*_ (%)	Min	Max
1	32.847 ± 11.928 0.0%	13.594	68.401	67.560 ± 23.797 0.0%	26.782	124.882	0.105 ± 0.046 0.0%	0.038	0.257
2	31.520 ± 10.901 3.8%	11.755	56.038	69.061 ± 23.641 3.0%	30.298	120.394	0.095 ± 0.039 9.0%	0.039	0.199
3	30.783 ± 11.880 6.1%	10.719	60.730	64.058 ± 22.609 4.4%	28.111	125.166	0.106 ± 0.041 1.6%	0.042	0.214
4	34.730 ± 11.006 5.9%	13.937	65.094	69.336 ± 21.368 3.4%	28.125	117.166	0.103 ± 0.045 1.6%	0.038	0.289
5	34.060 ± 9.390 3.8%	14.367	55.307	65.089 ± 19.183 2.8%	26.432	124.000	0.114 ± 0.044 8.7%	0.045	0.263
Group III	32.788 ± 11.115	10.719	68.401	67.021 ± 22.198	26.432	125.166	0.104 ± 0.043	0.038	0.289
